# Survival and predictive factors in dialysis patients with COVID-19 in Japan: a nationwide cohort study

**DOI:** 10.1186/s41100-021-00378-0

**Published:** 2021-10-21

**Authors:** Kan Kikuchi, Masaomi Nangaku, Munekazu Ryuzaki, Tomoyuki Yamakawa, Oota Yoshihiro, Norio Hanafusa, Ken Sakai, Yoshihiko Kanno, Ryoichi Ando, Toshio Shinoda, Hidetomo Nakamoto, Tadao Akizawa, COVID-19 Task Force Committee of the Japanese Association of Dialysis Physicians, the Japanese Society for Dialysis Therapy, and the Japanese Society of Nephrology

**Affiliations:** 1 Division of Nephrology, Shimoochiai Clinic, 2-1-6 Shimoochiai, Shinjuku-ku, Tokyo, 161-0033 Japan; 2 Division of Nephrology and Endocrinology, The University of Tokyo Graduate School of Medicine, Tokyo, Japan; 3 Department of Nephrology, Tokyo Saiseikai Central Hospital, Tokyo, Japan; 4 Kidney Center, Shirasagi Hospital, Osaka, Japan; 5 Nagoya Memorial Hospital, Nagoya, Japan; 6 Department of Blood Purification, Tokyo Women’s Medical University, Tokyo, Japan; 7 Department of Nephrology, Faculty of Medicine,, Toho University, Tokyo, Japan; 8 Department of Nephrology, Tokyo Medical University, Tokyo, Japan; 9 Department of Nephrology, Seishokai Memorial Hospital, Tokyo, Japan; 10 Faculty of Medical and Health Sciences, Tsukuba International University, Tsuchiura, Japan; 11 Department of General Internal Medicine, Saitama Medical University, Iruma, Japan; 12 Division of Nephrology, Department of Medicine, Showa University School of Medicine, Tokyo, Japan

**Keywords:** COVID-19, SARS-CoV-2, Dialysis, Peritoneal dialysis, Remdesivir

## Abstract

**Background:**

The Japanese Association of Dialysis Physicians, the Japanese Society for Dialysis Therapy, and the Japanese Society of Nephrology jointly established COVID-19 Task Force Committee and began surveying the number of newly infected patients.

**Methods:**

This registry of the COVID-19 Task Force Committee was used to collect data of dialysis patients; a total of 1010 dialysis patients with COVID-19 were included in the analysis. Overall survival of patients was investigated with stratification by age group, complication status, and treatment. In addition, predictive factors for mortality were also investigated. The overall survival was estimated by Kaplan–Meier methods and compared by using log-rank test. Multivariate analysis was performed to identify the risk factor of mortality. For all statistical analyses, *p* < 0.05 was considered to be statistically significant.

**Results:**

The mortality risk was increased with age (*p* < 0.001). The mortality risk was significantly higher in patients with peripheral arterial disease (HR: 1.49, 95% CI 1.05–2.10) and significantly lower in patients who were treated with remdesivir (HR: 0.60, 95% CI 0.37–0.98). Multivariate analysis showed increased risk of mortality with increment in BMI, and increment in CRP, and decreased risk with increment in albumin.

**Conclusion:**

Dialysis patients have a high severity of illness and a high risk of mortality in cases of COVID-19. Treatment with remdesivir might be effective in shortening the duration of hospitalization and reducing the risk of mortality.

## Background

In 2019, the new coronavirus disease (COVID-19) emerged from Wuhan, Hubei Province, China, and has rapidly spread around the world. The World Health Organization declared it to be a pandemic on March 11, 2020. As of August 14, 2021, there were 205,338,159 COVID-19 cases and 4,333,094 deaths worldwide [1].

In the general population of Japan, the first case of severe acute respiratory syndrome coronavirus 2 (SARS-CoV-2) was detected on January 15, 2020, in a patient with pneumonia who had traveled to Wuhan City. Since then, we have experienced a rapid increase in the number of new patients with COVID-19 from the first wave to the fifth wave, with a total of 1,108,269 COVID-19 cases and 15,383 deaths reported as of August 14, 2021 [2]. In the dialysis patients, on the other hand, the first patient with COVID-19 was reported on March 1, 2020. Soon after that, the Japanese Association of Dialysis Physicians, the Japanese Society for Dialysis Therapy, and the Japanese Society of Nephrology jointly established COVID-19 Task Force Committee to survey the number of newly infected patients and create guidance on preventive measures for COVID-19 for raising awareness [3]. The fifth wave began in Japan in July 2021, and a rapid increase in the number of newly infected dialysis patients was observed, with a cumulative total of 2156 infected dialysis patients as of August 12, 2021 [4].

The COVID-19 Task Force Committee summarized the infection situation among dialysis patients in Japan in 2020 and reported that severity and mortality rate were higher in the dialysis patients compared to that in the general population [3]. In this manuscript, we report the results of the risk factors of mortality and the effect of treatment in Japanese dialysis patients with COVID-19 up to the end of the fourth wave.

## Methods

### Subjects and data

Surveillance of new cases of COVID-19 in dialysis facilities in Japan was initiated by the COVID-19 Task Force Committee of the Japanese Association of Dialysis Physicians, the Japanese Society for Dialysis Therapy, and the Japanese Society of Nephrology on April 8, 2020 [3]. This registry was used to collect data of dialysis patients; data of a total of 1,948 dialysis patients with COVID-19 who were registered by June 19, 2021, were extracted. Among those, data of 897 patients (893 patients whose outcome was unknown and 4 patients whose age was unknown) were excluded, and a total of 1010 patients were included in this analysis.

Patient background data (age, gender, primary disease, duration of dialysis, complications, oxygenation, treatment for COVID-19) were collected; however, smoking status data were not collected. Blood test data at the time of diagnosis or hospitalization [albumin, blood urea nitrogen, creatinine, C-reactive protein (CRP), white blood cell count, hemoglobin, and platelet count] were available in patients who registered after March 16, 2021; these data were collected from a total of 311 patients whose blood test data were available. Treatment policy by the Ministry of Health, Labour and Welfare in Japan was implemented in which dialysis patients diagnosed with COVID-19 are treated with hospitalization [3].

Overall survival of patients was investigated with stratification by age group, complication status, and treatment. In terms of treatment for COVID-19, the efficacy of remdesivir was investigated among matched patients by using propensity score for age and oxygenation [with or without oxygen supplementation, ventilator, or extracorporeal membrane oxygenation (ECMO)] at the ratio of 1:3 for the patient group treated with remdesivir and the patient group not treated with remdesivir. The duration of hospitalization was also compared between the patient group treated with remdesivir and the patient group not treated with remdesivir. In terms of dialysis, overall survival was compared between patients who underwent peritoneal dialysis and those who underwent hemodialysis matched using the propensity score for age and oxygenation (with or without oxygen supplementation, ventilator, or ECMO) at the ratio of 1:3.

### Statistical analysis

Categorical data were analyzed using Fisher’s exact test, and continuous data were analyzed using Welch’s *t* test or Mann–Whitney’s U-test. For survival analysis, the survival probability was estimated by Kaplan–Meier methods and compared using log-rank test. The multiplicity was adjusted by Bonferroni method. Hazard ratios and associated 95% confidence intervals were assessed by Cox regression hazard model.

The univariate and multivariate analyses were performed to identify the risk factor of mortality, with incidence of COVID-19 in facilities (less than 5 or more than 5), age (< 60, 60 s, or ≥ 70), gender, primary disease (chronic glomerulonephritis, diabetes mellitus, nephrosclerosis, or others), duration of dialysis (< 1 year, 1 to < 5 years, 5 to < 10 years, 10 to < 15 years, or ≥ 15 years), complications (diabetes mellitus, hypertension, cardiovascular disease, peripheral arterial disease, or malignancy), oxygenation (with or without oxygen supplementation, ventilator, or ECMO), treatment for COVID-19 (with or without remdesivir or dexamethasone) as independent variables. The univariate and multivariate analyses were performed to identify the risk factors of mortality also in those who had blood test data at the time of diagnosis or hospitalization, with age (< 60, 60 s, or ≥ 70), gender, primary disease (chronic glomerulonephritis, diabetes mellitus, nephrosclerosis, or others), duration of dialysis (< 1 year, 1 to < 5 years, 5 to < 10 years, 10 to < 15 years, or ≥ 15 years), BMI, albumin, blood urea nitrogen, creatinine, CRP, white blood cell count, hemoglobin, and platelet count as independent variables.

All analyses were performed using SPSS Statistics version 21 (IBM SPSS Statistics for Windows, IBM, Armonk, NY), and *p* < 0.05 was considered to be statistically significant. This study was approved by the Ethics Committee of the Japanese Society for Dialysis Therapy (authorization number: 1–8), and all procedures adhered to the Declaration of Helsinki.

## Results

### Comparison of patient background between patient groups who recovered and who died

The patient background and blood test data of patient groups of those who were recovered and those who died are shown in Tables 1 and 2, respectively. Among 1010 patients included in this analysis, 699 patients (69.2%) recovered and 311 patients (30.8%) died. The age was higher and duration of dialysis was longer in the patient group who died; however, there was no difference in gender or primary disease for induction of dialysis between groups. In terms of complications, the proportions of patients with cardiovascular disease and peripheral arterial disease were higher in the patient group who died. Moreover, the proportion of patients who had oxygenation, or treated with dexamethasone was higher in the patient group who died. Among 311 patients whose blood test data were available, body mass index (BMI), creatinine, and albumin were lower and CRP was higher in the patient group who died.

**Table 1:** Background of patients

	Recovered		Died		*p* value^a^
	*n*	%	*n*	%	
Age					
< 60	250	35.8	29	9.3	< 0.001
60 s	164	23.5	45	14.5	
≥ 70	285	40.8	237	76.2	
Gender					
Male	497	71.3	212	68.4	0.37
Female	200	28.7	98	31.6	
Primary disease					
Chronic glomerulonephritis	123	19.4	37	13.8	0.211
Diabetes mellitus	328	51.8	147	54.6	
Nephrosclerosis	87	13.7	43	16.0	
Others	95	15.0	42	15.6	
Duration of dialysis					
< 1 year	95	13.9	21	7.5	0.015
1 to < 5 years	257	37.6	94	33.7	
5 to < 10 years	164	24.0	78	28.0	
10 to < 15 years	83	12.1	45	16.1	
≥ 15 years	85	12.4	41	14.7	
Complication					
Hypertension					
No	383	56.2	158	57.0	0.83
Yes	299	43.8	119	43.0	
Diabetes mellitus					
No	335	48.4	120	42.7	0.119
Yes	357	51.6	161	57.3	
Cardiovascular disease					
No	420	62.5	131	48.9	< 0.001
Yes	252	37.5	137	51.1	
Chronic respiratory disease					
No	625	92.5	243	89.3	0.122
Yes	51	7.5	29	10.7	
Peripheral arterial disease					
No	585	87.3	198	74.7	< 0.001
Yes	85	12.7	67	25.3	
Malignancy					
No	586	86.8	226	84.0	0.298
Yes	89	13.2	43	16.0	
Number of complications					
0	114	16.5	29	10.2	0.008
1	218	31.5	80	28.2	
≥ 2	361	52.1	175	61.6	
Oxygenation					
No	302	44.8	29	10.5	< 0.001
Yes	320	47.5	174	63.0	
Ventilator or ECMO	52	7.7	73	26.4	
Remdesivir					
No	591	89.0	235	90.0	0.723
Yes	73	11.0	26	10.0	
Dexamethasone					
No	374	56.2	107	40.5	< 0.001
Yes	291	43.8	157	59.5	

*ECMO* extracorporeal membrane oxygenation

^a^Fisher’s exact test

**Table 2:** BMI and blood test data of patients

	Recovered	Died	*p* value
BMI (kg/m^2^)			
*n*	197	100	0.01^a^
Mean ± SD	23.5 ± 5.3	22.0 ± 4.6	
Alb (g/dL)			
*n*	204	65	< 0.001^a^
Mean ± SD	3.3 ± 0.6	2.9 ± 0.6	
BUN (mg/dL)			
*n*	208	94	0.018^a^
Mean ± SD	56.4 ± 19.7	64.2 ± 28.8	
Cr (mg/dL)			
*n*	208	94	0.004^a^
Mean ± SD	10.1 ± 4.1	8.8 ± 3.5	
CRP (mg/dL)			
*n*	202	92	< 0.001^b^
Mean (IQR)	2.0 (0.6–6.2)	7.1 (3.0–12.8)	
WBC (/μL)			
*n*	213	97	0.001^b^
Mean (IQR)	5150 (4000–6600)	6600 (4100–8920)	
Hb (g/dL)			
*n*	214	96	0.775^a^
Mean (IQR)	11.2 ± 2.7	11.1 ± 1.5	
PLT (万/μL)			
*n*	214	97	0.018^b^
Mean (IQR)	19.3 ± 26.6	21.2 ± 38.1	

*BMI* body mass index, *Alb* albumin, *BUN* urea nitrogen, *Cr* creatinine, *CRP* C-reactive protein, *WBC* white blood cell count, *Hb* hemoglobin, *PLT* platelet count, *SD* standard deviation, *IQR* interquartile range

^a^Welch’s *t* test

^b^Mann–Whitney's U-test

### Survival of patients stratified by age group, complication status, and treatment for COVID-19

Comparison of overall survival of patients stratified by age group (< 60, 60 s, or ≥ 70) showed that the mortality risk was increased with age (*p* < 0.001) (Fig. 1). According to the univariate analysis, the mortality risk was significantly higher in the patient group with age 60 s [hazard ratio (HR): 2.02, 95% confident interval (CI) 1.27–3.23)] and in the patient group with age ≥ 70 (HR: 3.13, 95% CI 3.13–6.77) when comparing to the patient group with age < 60. According to the multivariate analysis, the mortality risk was significantly higher in the patient group with age ≥ 70 (HR: 4.92, 95% CI 3.10–7.80) but not in the patient group with age 60 s (HR: 1.58, 95% CI 0.90–2.77) when comparing to the patient group with age < 60 (Table 3).

**Fig. 1:** Overall survival stratified by age groups (< 60, 60 s, and ≥ 70)

**Table 3:** Multivariate analysis on predictive factors for mortality

	Hazard ratio	95% confidence interval of hazard ratio		*p* value
		Lower limit	Upper limit	
Age (reference: < 60)				
60 s	1.58	0.90	2.77	0.109
≥ 70	4.92	3.10	7.80	< 0.001
Gender (reference: male)	0.82	0.60	1.11	0.202
Primary disease (reference: chronic glomerulonephritis)				
Diabetes mellitus	1.16	0.46	2.95	0.751
Nephrosclerosis	0.94	0.55	1.61	0.829
Others	1.56	0.91	2.68	0.106
Duration of dialysis (reference: < 1 year)				
1 to < 5 years	2.07	1.21	3.53	0.008
5 to < 10 years	2.00	1.16	3.45	0.013
10 to < 15 years	2.69	1.49	4.85	0.001
≥ 15 years	2.68	1.48	4.88	0.001
Complication				
Diabetes mellitus	1.12	0.45	2.77	0.813
Hypertension	0.87	0.65	1.16	0.337
Cardiovascular disease	1.25	0.94	1.68	0.130
Chronic respiratory disease	0.87	0.55	1.38	0.561
Peripheral arterial disease	1.49	1.05	2.10	0.025
Malignancy	0.91	0.62	1.33	0.626
Oxygenation (reference: no oxygenation)				
Oxygen supplementation	3.44	2.06	5.73	< 0.001
Ventilator or ECMO	6.72	3.86	11.69	< 0.001
Remdesivir (reference: without remdesivir)	0.60	0.37	0.98	0.041
Dexamethasone (Reference: without dexamethasone)	1.36	1.01	1.83	0.040

Multivariate analysis was performed, with incidence of COVID-19 in facilities (less than 5 or more than 5), age (< 60, 60 s, ≥ 70), gender, primary disease (chronic glomerulonephritis, diabetes mellitus, nephrosclerosis, or others), duration of dialysis (< 1 year, 1 to < 5 years, 5 to < 10 years, 10 to < 15 years, or ≥ 15 years), complications (diabetes mellitus, hypertension, cardiovascular disease, peripheral arterial disease, or malignancy), oxygenation (with or without oxygen supplementation, ventilator, or ECMO), treatment for COVID-19 (with or without remdesivir or dexamethasone) as independent variables

*ECMO* extracorporeal membrane oxygenation

The multivariate analysis also showed significant increase in mortality with prolonging duration of dialysis; however, there was no difference in gender or primary disease. The mortality risk was significantly higher in patients with peripheral arterial disease (HR: 1.49, 95% CI 1.05–2.10) in terms of complication and was significantly lower in patients who were treated with remdesivir (HR: 0.60, 95% CI 0.37–0.98) in terms of treatment for COVID-19 (Table 3).

### Efficacy of remdesivir

A total of 392 patients were analyzed (98 patients who were treated with remdesivir and matched 294 patients who were not treated with remdesivir); the background of those patients is shown in Table 4. The overall survival was significantly prolonged in the patient group who were treated with remdesivir than in the patient group who were not treated with remdesivir (HR: 0.45, 95% CI 0.26–0.80, *p* = 0.004) (Fig. 2). Moreover, the duration of hospitalization (mean ± standard deviation) was 20.9 ± 13.2 days in the patient group who were treated with remdesivir, which was significantly shorter than 16.2 ± 8.1 days in the patient group who were not treated with remdesivir (Difference: 4.7 days, 95% CI 2.2–7.4, *p* < 0.001).

**Table 4:** Background of patients stratified by administration of remdesivir (with or without remdesivir) after matching

	Without remdesivir		With remdesivir		*p* value^a^
	*n*	%	*n*	%	
Age					
< 60	90	30.6	30	30.6	1.000
60 s	51	17.3	17	17.3	
≥ 70	153	52.0	51	52.0	
Gender					
Male	210	71.7	67	68.4	0.524
Female	83	28.3	31	31.6	
Primary disease					
Chronic glomerulonephritis	40	15.1	20	22.5	0.372
Diabetes mellitus	149	56.2	43	48.3	
Nephrosclerosis	39	14.7	12	13.5	
Others	37	14.0	14	15.7	
Duration of dialysis					
< 1 year	37	12.9	14	14.4	0.754
1 to < 5 years	100	34.8	31	32.0	
5 to < 10 years	72	25.1	30	30.9	
10 to < 15 years	42	14.6	13	13.4	
≥ 15 years	36	12.5	9	9.3	
Complication					
Hypertension					
No	156	55.1	42	42.9	0.046
Yes	127	44.9	56	57.1	
Diabetes mellitus					
No	124	43.5	46	46.9	0.558
Yes	161	56.5	52	53.1	
Cardiovascular disease					
No	156	56.5	49	51.6	0.406
Yes	120	43.5	46	48.4	
Chronic respiratory disease					
No	249	89.6	83	87.4	0.571
Yes	29	10.4	12	12.6	
Peripheral arterial disease					
No	230	84.9	75	78.9	0.201
Yes	41	15.1	20	21.1	
Malignancy					
No	234	84.2	83	87.4	0.509
Yes	44	15.8	12	12.6	
Number of complication					
0	38	13.1	10	10.2	0.778
1	84	29.1	29	29.6	
≥ 2	167	57.8	59	60.2	
Oxygenation					
No	69	23.5	23	23.5	1.000
Yes	159	54.1	53	54.1	
Ventilator or ECMO	66	22.4	22	22.4	

*ECMO* extracorporeal membrane oxygenation

^a^Fisher’s exact test

**Fig. 2:** Overall survival stratified by administration of remdesivir (with or without remdesivir)

### Predictive factors for mortality

A total of 311 patients whose blood test data were available were analyzed. Among those patients, BMI was lower in the patient group who died. Multivariate analysis showed that the risk of mortality was increased with every 1 increment in BMI (HR: 1.10, 95% CI 1.01–1.19). The risk of mortality was also increased with every 1 increment in CRP (HR 1.26, 95% CI 1.01–1.56). On the other hand, the risk of mortality was decreased with every 1 increment in albumin (HR 0.48, 95% CI 0.24–0.97) (Table 5).

**Table 5:** Multivariate analysis on predictive factors for mortality

	Hazard ratio	95% confidence interval of hazard ratio		*p* value
		Lower limit	Upper limit	
Age (reference: < 60)				
60 s	2.73	0.96	7.79	0.061
≥ 70	6.03	1.98	18.42	0.002
Gender (reference: male)	0.60	0.29	1.26	0.177
Primary disease (reference: chronic glomerulonephritis)				
Diabetes mellitus	1.08	0.46	2.54	0.866
Nephrosclerosis	1.76	0.60	5.12	0.302
Others	1.87	0.60	5.85	0.280
Duration of dialysis (reference: < 1 year)				
1 to < 5 years	8.99	1.06	76.15	0.044
5 to < 10 years	9.65	1.16	80.44	0.036
10 to < 15 years	21.91	2.15	223.26	0.009
≥ 15 years	22.76	2.50	207.23	0.006
Data				
BMI	1.10	1.01	1.19	0.021
Alb	0.48	0.24	0.97	0.040
BUN	1.02	1.00	1.04	0.039
Cr	0.91	0.79	1.04	0.166
CRP (log)	1.26	1.01	1.56	0.041
WBC (log)	1.54	0.87	2.73	0.137
Hb	1.06	0.87	1.30	0.565
PLT (log)	1.09	0.66	1.82	0.730

Multivariate analysis was performed, with age (< 60, 60 s, or ≥ 70), gender, primary disease (chronic glomerulonephritis, diabetes mellitus, nephrosclerosis, others), duration of dialysis (< 1 year, 1 to < 5 years, 5 to < 10 years, 10 to < 15 years, or ≥ 15 years), BMI, albumin, blood urea nitrogen, creatinine, CRP, white blood cell count, hemoglobin, and platelet count as independent variables

All data show hazard ratio for every 1 increase in value

*BMI* body mass index, *Alb* albumin, *BUN* blood urea nitrogen, *Cr* creatinine, *CRP* C-reactive protein, *WBC* white blood cell count, *Hb* hemoglobin, *PLT* platelet count

### Overall survival in patients who underwent peritoneal dialysis or hemodialysis

A total of 100 patients (25 patients in the patient group who underwent peritoneal dialysis and 75 patients in the patient group who underwent hemodialysis) were analyzed; the patients background is shown in Table 6. Four deaths (20.0%) were reported in the patient group who underwent peritoneal dialysis, while 16 deaths (21.3%) were reported in the patient group who underwent hemodialysis. The overall survival was not significantly different between the patient groups who underwent peritoneal dialysis and those who underwent hemodialysis (*p* = 0.3) (Fig. 3). The overall survival was not significantly different in the patient group who underwent peritoneal dialysis compared to that in the patient group who underwent hemodialysis (HR: 0.61, 95% CI 0.23–1.63). The duration of hospitalization (mean ± standard deviation) was 18.1 ± 9.9 days in the patient group who underwent peritoneal dialysis compared to 18.0 ± 10.0 days in the patient group who underwent hemodialysis; there was no significant difference between the groups (*p* = 0.96).

**Table 6:** Background of patients stratified by dialysis treatment (peritoneal dialysis or hemodialysis) after matching

	Hemodialysis		Peritoneal dialysis		*p* value^a^
	*n*	%	*n*	%	
Age					
< 60	36	48.0	12	48.0	1.000
60 s	21	28.0	7	28.0	
≥ 70	18	24.0	6	24.0	
Gender					
Male	55	73.3	20	80.0	0.601
Female	20	26.7	5	20.0	
Primary disease					
Chronic glomerulonephritis	15	21.1	8	36.4	0.507
Diabetes mellitus	36	50.7	8	36.4	
Nephrosclerosis	6	8.5	2	9.1	
Others	14	19.7	4	18.2	
Duration of dialysis					
< 1 year	10	13.7	6	24.0	0.032
1 to < 5 years	24	32.9	14	56.0	
5 to < 10 years	22	30.1	5	20.0	
10 to < 15 years	9	12.3	0	0.0	
≥ 15 years	8	11.0	0	0.0	
Complication					
Hypertension					
No	41	54.7	12	50.0	0.815
Yes	34	45.3	12	50.0	
Diabetes mellitus					
No	36	48.0	16	66.7	0.159
Yes	39	52.0	8	33.3	
Cardiovascular disease					
No	51	69.9	21	87.5	0.110
Yes	22	30.1	3	12.5	
Chronic respiratory disease					
No	67	91.8	24	100.0	0.331
Yes	6	8.2	0	0.0	
Peripheral arterial disease					
No	64	87.7	23	95.8	0.443
Yes	9	12.3	1	4.2	
Malignancy					
No	65	90.3	23	95.8	0.675
Yes	7	9.7	1	4.2	
Number of complications					
0	12	16.0	6	25.0	0.164
1	25	33.3	11	45.8	
≥ 2	38	50.7	7	29.2	
Oxygenation					
No	12	16.0	4	16.0	1.000
Yes	54	72.0	18	72.0	
Ventilator or ECMO	9	12.0	3	12.0	
Remdesivir					
No	63	87.5	23	95.8	0.443
Yes	9	12.5	1	4.2	
Dexamethasone					
No	27	37.5	11	45.8	0.481
Yes	45	62.5	13	54.2	

^a^Fisher’s exact test

**Fig. 3:** Overall survival stratified by dialysis treatment (peritoneal dialysis or hemodialysis)

## Discussion

Our study showed that the mortality rate among dialysis patients in Japan was high at 30.8%, which was 20 times higher than the mortality rate of 1.5% in the general population for the same period, June 16, 2021 [5]. The mortality rate of dialysis patients by age group was 10.4% for those under 60, 21.5% for those in their 60 s, and 45.4% for those over 70, while the mortality rate in the general population was 0.07% for those under 60, 1.3% for those in their 60 s, and 9.1% for those over 70, indicating a very high mortality rate for dialysis patients in all age groups [5]. However, Japan is not the only country with a high mortality rate among dialysis patients, and the data were similar to those in the USA and results of meta-analysis [6, 7]. The factors associated with increased risk of mortality were identified as aged over 70, having a long duration of dialysis, need of oxygenation, high CRP in laboratory data at diagnosis, high BMI, and complication of peripheral arterial disease. In a report on dialysis patients in the USA, complication of peripheral arterial disease was identified as an important risk factor [6]. In addition, hypercoagulation and vascular damage have been reported to be involved in the pathogenesis of COVID-19 [8], and thrombosis and elevated inflammatory response with CRP have been reported to be associated with worsening of symptoms [9–11]. Dialysis patients with peripheral arterial disease often have concomitant systemic vascular disease and small artery disease, which might lead to increase the risk of mortality.

The results showed that the risk of mortality decreased as the albumin level increased. Since nutrition is an important factor related to immunity, and increase in CRP and complication of peripheral arterial disease are risk factors of mortality, malnutrition, inflammation, and atherosclerosis syndrome (MIA syndrome) known to occur in dialysis patients [12, 13] might lead to risk of increasing the severity of COVID-19 and mortality.

The mortality rate of patients with peritoneal dialysis was 16.0% (4/25 patients), which is lower than 25% (2/8 patients) in China [14] and 18.2% (2/11 patients) in the USA [15]; however, caution is needed to interpret these data due to small sample size. In Japan, the mortality risk was compatible among patients who underwent peritoneal dialysis and matched those who underwent hemodialysis, which might be because all dialysis patients diagnosed with COVID-19 were treated with hospitalization.

As for the prevalence rate of COVID-19, since the number of dialysis patients in Japan in 2020 and 2021 has not been reported yet, the calculation using the data as of December 31, 2019 [16] shows a lower prevalence rate of 0.25% (25/9746) in peritoneal dialysis compared to 0.57% (1.948/344,640) in all dialysis patients. However, statistical analysis cannot be performed since the total number of dialysis patients at the time of COVID-19 occurrence (denominator) is unknown. The prevalence of a study of 810 patients with peritoneal dialysis in Wuhan, China, was reported to be 2.44/1000 person-months [14], which is similar to that in patients with peritoneal dialysis in Japan.

Although the United States Food and Drug Administration (FDA) does not recommend remdesivir for patients with eGFR < 30 mL/min/1.73 m^2^, the safety and tolerability of remdesivir were investigated in 48 dialysis patients with COVID-19 by Aiswarya et al. [17]. The results showed that the duration of hospitalization was shortened by an average of 5.5 days in the patients who received remdesivir within 48 h of hospitalization compared to those who did not receive remdesivir within 48 h of hospitalization (*p* = 0.001), and the safety of remdesivir was also confirmed. Our study results with the propensity score matching demonstrated that duration of hospitalization was shortened by 4.7 days in the patients who received remdesivir compared to those who did not (*p* < 0.001). Moreover, the overall survival was significantly prolonged in the patients who received remdesivir compared to that in patients who did not receive remdesivir [HR: 0.45 (95% CI 0.26–0.80)]. Remdesivir was confirmed to be an effective treatment option for dialysis patients in Japan.

In the case of COVID-19, the severity of the disease in dialysis patients is high and the risk of mortality is also high. Thus, it is important to take infection control measures to prevent the infection of SARS-CoV-2, and the COVID-19 Task Force Committee has been promoting awareness of infection control measures [18]. In addition, prevention of infection, onset of disease, and prevention of severe symptoms through vaccination are important. According to the surveillance of the COVID-19 Task Force Committee, the prevalence ratio of dialysis patients to the general population has decreased since 1 month after the vaccination in the elderly population aged over 65 years was started in Japan. In the third wave, December 2020 and January 2021, there were 235,800 new cases were reported in the general population, while 720 new cases were reported in dialysis patients; the prevalence rate was 1 per 328 in the general population. However, in the fourth wave, May and June 2021, there were 225,006 new cases were reported in the general population and 330 new cases were reported in dialysis patients; the prevalence rate was 1 per 682 in the general population. This is thought to be due to the fact that the majority of dialysis patients had vaccination early since the proportion of population of dialysis patients aged over 65 years is twice as large as population of the general population aged over 65 years [18].

## Conclusion

In conclusion, dialysis patients have a high severity of illness and a high risk of mortality in cases of COVID-19. Therefore, awareness and implementation of infection control measures are important. Treatment with remdesivir might be effective in shortening the duration of hospitalization and reducing the risk of mortality.

## Data Availability

None.

## Abbreviations

BMI: Body mass index
COVID-19: New coronavirus disease
CRP: C-reactive protein
ECMO: Extracorporeal membrane oxygenation
SARS-CoV-2: Severe acute respiratory syndrome coronavirus 2
